The article "Combination of total glucosides of paeony, narrow‐band ultraviolet B, and oral corticosteroid mini‐pulse therapy for nonsegmental vitiligo: A retrospective study" was published in 2024. Journal: Skin Res Technol.

# Combination of total glucosides of paeony, narrow‐band ultraviolet B, and oral corticosteroid mini‐pulse therapy for nonsegmental vitiligo: A retrospective study

**DOI:** 10.1111/srt.13769

**Published:** 2024-06-17

**Authors:** Jiachen Gui, Zhimin Li, Bin Zhou, Qiang Li, Yue Zhang, Yaojun Wang, Jiaoni Chi, Tao Wang

**Affiliations:** ^1^ Graduate School Air Force Medical University Xi'an P. R. China; ^2^ Department of Dermatology Air Force Medical Center, PLA Beijing P. R. China; ^3^ Graduate School Hebei North University Zhangjiakou P. R. China; ^4^ Handan Second Hospital Handan P. R. China; ^5^ Department of Allergy State Key Laboratory of Complex Severe and Rare Diseases Peking Union Medical College Hospital, Chinese Academy of Medical Science and Peking Union Medical College Beijing P. R. China; ^6^ Department of Dermatology West China Hospital, Sichuan University Chengdu P. R. China

**Keywords:** retrospective study, total glucoside of paeony, traditional Chinese medicine, vitiligo

## Abstract

**Background:**

The total glucoside of paeony (TGP) is recognized for its immunomodulatory properties and anti‐inflammatory effects. This study evaluates the efficacy of TGP combined with oral mini‐pulse therapy (OMP) and narrow‐band ultraviolet B (NB‐UVB) in treating active nonsegmental vitiligo (NSV).

**Materials and methods:**

The combination therapy was contrasted against those from a group treated solely with OMP and NB‐UVB. Data from 62 patients undergoing TGP combination treatment and 55 without were analyzed over a 3‐month period. After 6 months, the differences in recurrence rate were investigated by follow‐up.

**Results:**

The findings indicate that integrating TGP may yield superior outcomes compared to OMP + NB‐UVB alone. Moreover, the patient's oxidative stress makers were significantly reduced after the treatment. The majority of patients in the TGP cohort exhibited enhanced skin pigmentation over the duration. Notably, no increase in side effects or recurrence was observed in this group. Especially, patients with vitiligo on their head and neck experienced pronounced improvements.

**Conclusion:**

The efficacy of the combination treatment group was better than that of the control group at 2 and 3 months, and there was no difference in recurrence rate and side effects, suggesting that TGP may continue to show efficacy in NSV for a longer period of time by reducing the level of oxidative stress, and is especially suitable for patients with head and neck lesions.

## 1 INTRODUCTION

Within traditional Chinese medicine (TCM), the total glucoside of paeony (TGP) holds a significant place, with references in classical Chinese medical texts dating between 475 and 221 BCE.^1^ Modern science identifies Paeoniflorin (PF) as TGP's primary active component.^2^ TGP has demonstrated robust anti‐inflammatory and immunomodulatory effects, complemented by its antioxidant capabilities.^3^, ^4^, ^5^, ^6^ Consequently, while much of TGP research has focused on inflammatory conditions, its potential in vitiligo treatment remains largely unexplored. Yu et al. found that PF markedly reduced ROS formation within EA.hy926 cells, attenuated malondialdehyde (MDA) and lactate dehydrogenase (LDH) release, and augmented the synthesis of endogenous antioxidants such as glutathione (GSH) and superoxide dismutase (SOD).^7^ A study by Yuan et al. elucidated TGP's mechanistic role in melanocyte protection against oxidative stress. Using PIG1 and PIG3V cell lines, the research indicated PF pretreatment elevated antioxidant enzyme activity, notably SOD and catalase (CAT), with the JNK/Nrf2/HO‐1 signaling pathway strengthening cellular defenses against oxidative distress.^8^ An animal study highlighted that PF treatment at 10 µg/mL significantly promoted melanin synthesis in melanocytes and increased protein concentrations of microphthalmia‐associated transcription factor (MITF) and tyrosinase‐related protein 1 (TRP‐1). Additionally, it augmented the phosphorylation of cAMP‐response element binding (CREB) and extracellular signal‐regulated kinase (ERK), implying its effect through the ERK/CREB pathway. Moreover, paeoniflorin demonstrated effectiveness in reducing vitiligo symptoms in mice.^9^ Consequently, paeoniflorin is posited as a prospective therapeutic agent for vitiligo, paving the way for subsequent clinical research on its influence on the condition.

The article "Combination of total glucosides of paeony, narrow‐band ultraviolet B, and oral corticosteroid mini‐pulse therapy for nonsegmental vitiligo: A retrospective study" was published in 2024. Journal: Skin Res Technol.

Vitiligo is a prevalent skin pigmentation disorder, affecting approximately 0.5%–2% of the global population.^10^ A leading hypothesis attributes its onset to oxidative stress, wherein reactive oxygen species (ROS) facilitate melanocyte degradation through complex pathways such as JNK/Nrf2/HO‐1.^11^ Predominantly, nonsegmental vitiligo (NSV) constitutes the major form, accounting for an astonishing 80%−90% of all diagnosed cases.^12^ Presently, vitiligo treatments encompass a wide range of approaches, including topical and oral steroids, along with advanced methods such as phototherapies.^13^

In recent times, the combination of systemic corticosteroids (CSs) with narrow‐band UVB (NB‐UVB) has emerged as a promising treatment strategy.^14^ Nonetheless, due to a range of side effects, the utilization of CSs is often relegated to a secondary role. Conversely, oral mini‐pulse therapy (OMP) is garnering attention owing to its favorable safety‐efficacy profile.^15^ Clinical trials have highlighted the enhanced efficacy of combining OMP with NB‐UVB, indicating potential advantages over singular treatments; utilizing OMP + NB‐UVB for vitiligo facilitated significant improvement in 37.03% of patients and moderate improvement in 44.44% of patients, a marked progression compared to the 5 and 10% improvement observed with OMP alone.^16^ Numerous other studies have corroborated these findings.^17^, ^18^

This study explores the potential outcomes of incorporating TGP with established NSV treatments. By conducting an extensive retrospective analysis, we aim to delineate the therapeutic effectiveness of a TGP, OMP, and NB‐UVB amalgamation in mitigating active NSV. Simultaneously, we seek to identify potential discrepancies in treatment outcomes across different anatomical regions.

The article "Combination of total glucosides of paeony, narrow‐band ultraviolet B, and oral corticosteroid mini‐pulse therapy for nonsegmental vitiligo: A retrospective study" was published in 2024. Journal: Skin Res Technol.

## 2 MATERIAL AND METHODS

This study predominantly utilized case records from patients diagnosed with vitiligo who sought consultations at the Air Force Medical Center, PLA, in the year 2020. Our approach, especially with regards to active NSV patient selection, was heavily influenced by the comprehensive guidelines stipulated by the European Dermatology Forum consensus.^19^

### 2.1 Inclusion criteria

Gender: No restrictions were imposed based on gender, thus fostering a diverse patient pool. Disease activity: Only individuals exhibiting active NSV were selected, characterized by the emergence of fresh skin lesions within the past 6 months. Laboratory examinations: The patients were examined before and after treatment for complete blood count, biochemical tests, plasma electrolyte tests, and indicators of oxidative stress. Treatment consistency: Participants were required to adhere to a consistent regimen, accompanied by monthly evaluations to assess therapeutic efficacy. Post‐treatment observation: Following treatment completion, patients underwent a rigorous follow‐up period to monitor potential disease recurrences.

### 2.2 Exclusion criteria

Individuals who had utilized vitiligo‐specific topical medications within 2 weeks or engaged in systemic medication courses or phototherapy sessions for vitiligo within 4 weeks preceding the initial data collection were excluded.

As shown in Figure 1, from an extensive pool of 500 vitiligo patients, we screened 320 patients with active NSV. A further analysis of treatment methods revealed that 62 patients received a TGP‐related treatment regimen, these patients had received at least one previous treatment, including phototherapy and topical drug therapy, but were not satisfied with the results, so the new method was selected. All these patients were treated with TGP, OMP, and NB‐UVB for 3 months. We then selected 55 patients treated with OMP and NB‐UVB for 3 months as a control group. The treatment period is short because during the Corona Virus Disease 2019 (COVID‐19) pandemic, China's epidemic control measures are very strict, these patients were subjected to urban control policies after only 3 months of treatment, unable to travel to any hospital. Fortunately, patient compliance was not compromised during the 3‐month period. The whole city control policy did not end until 6 months later, we, therefore, analyzed the relapse rate at month 6 after the final treatment.

The article "Combination of total glucosides of paeony, narrow‐band ultraviolet B, and oral corticosteroid mini‐pulse therapy for nonsegmental vitiligo: A retrospective study" was published in 2024. Journal: Skin Res Technol.

**FIGURE 1:** The flow chart for patient inclusion.

Our study was approved by the ethics review board of the Air Force Medical Center, Air Force Medical University, People's Republic of China (2022‐50‐YJ01). Prior to initiating the study, our team established comprehensive communication with potential participants, soliciting their consent to use their medical data for research, with stringent assurances pertaining to data confidentiality and the nondisclosure of personal identifiers. The solicitation received an overwhelmingly positive response, securing unanimous consent from the approached patients, and they all signed informed consent forms.

Methylprednisolone Tablets (Medrol®, Pfizer Pharmaceuticals Ltd, Localita` Marino del Tronto, Ascoli Piceno, Italy), selected as the OMP agent, were characterized by its distinctive lipid‐soluble methyl compound, enhancing its efficiency as a medium‐acting glucocorticoid due to its inherent potassium‐retaining properties. This medication was administered at a dosage of 0.5 mg/kg over two successive days weekly. Concurrently, participants were prescribed Total Glucoside of White Paeony Capsules (Pafulin®, Ningbo Liwah Pharmaceutical Co., Ltd, Ningbo, Zhejiang Province, People's Republic of China) at a daily dosage of 0.6 g. Take it in three doses. The NB‐UVB treatment was administered by UV light therapy device (UV light therapy device SS‐10, Shanghai SIGMA hi‐tech Co., LTD, Shanghai, People's Republic of China), three times a week on nonconsecutive days. Before the commencement of the treatment, the minimum erythema dose (MED) for each patient was rigorously assessed. The initial dose was set at 70% of the patient's MED, with subsequent adjustments in increments of 10%–20%, not exceeding a ceiling of 3.0 J/cm^2^. This escalation protocol continued until erythema consistently appeared for a period ranging from 24 to 72 h. Following each session, the dose and duration of exposure were precisely documented. During the irradiation of the head and face, safety measures such as wearing protective eyewear were employed, and patients were instructed to firmly close their eyes.

The article "Combination of total glucosides of paeony, narrow‐band ultraviolet B, and oral corticosteroid mini‐pulse therapy for nonsegmental vitiligo: A retrospective study" was published in 2024. Journal: Skin Res Technol.

At the outset of the study, committed personnel were tasked with methodically documenting pertinent patient data. This data was later consolidated into structured tables for straightforward reference. Anticipating the potential challenges posed by confounding bias, we engaged our researchers in intensive training sessions, accentuating the importance of accuracy during data collection.

### 2.3 Statistics

After the preliminary organization of the experimental data using Excel 2010, we conducted statistical analyses utilizing the SPSS 26.0 software. The categorical data were scrutinized using the chi‐square test, while the normality of the continuous data underwent evaluation. Continuous data adhering to a normal distribution were denoted as “x ± s,” whereas data not following a normal distribution were represented using median and interquartile ranges, denoted as M (P25∼P75). We applied an independent sample *t*‐test to compare two groups with normally distributed data. In contrast, the Mann–Whitney *U* test served to analyze groups with data not following a normal distribution. Furthermore, the Kruskal–Wallis test facilitated the assessment of efficacy across various sites, succeeded by detailed pair‐wise comparisons. For bivariate correlation analysis, Pearson's correlation coefficient was used for data obeying normal distribution, and Spearman's correlation coefficient was used for ranked variables. We considered a *P*‐value <0.05 to indicate statistical significance.

## 3 RESULTS

Table 1 illustrates the demographic profile of the participants, whose ages ranged from 15 to 57 years, and the duration of their condition fluctuated between 1 and 252 months. To delineate the variances in the severity of the disease between the two groups, we used VASI scores for the assessment of baseline information.

**TABLE 1:** Demographic data of the two groups.

	Group		*X* ^2^/*Z*/*t*	*P*
	Case	Control		
Sex (%)				
Male	25(40.32)	27(49.09)	0.908	0.341
Female	37(59.68)	28(50.91)		
Age, mean ± SD (years)	24.56 ± 8.824	23.35 ± 9.27	0.728	0.468
Course, MD (months)	16.5(6, 32.25)	11(6, 25)	−1.092	0.275
Clinical typing (%)				
Acrofacial(acral)	20(32.26)	18(32.73)	0.007	0.997
Acrofacial(facial)	23(37.1)	20(36.36)		
Generalized	19(30.65)	17(30.91)		
VASI, mean ± SD	5.75 ± 2.89	4.86 ± 2.73	1.709	0.900

*Note*: *P*‐value < 0.05 considered as significant.

Abbreviations: MD, median; SD, standard deviation.

The baseline data confirmed that there were no significant differences in terms of gender, age, course, clinical typing, or VASI scores between the two groups.

Throughout the monthly evaluations, improvements were assessed by juxtaposing the current data with the baseline metrics, facilitating the determination of the repigmentation rate. We aligned our grading system with methodologies from Lee et al.’s research: Grade 1: 0%–25% repigmentation. Grade 2: 26%−50%. Grade 3: 51%−75%. Grade 4: 76%−90%. Grade 5: 91%−100%.^20^ The three‐month pigmentation grade analysis is shown in Table 2, and the specific percentage of patients with each grade in each month is more clearly described in Table 3.

The article "Combination of total glucosides of paeony, narrow‐band ultraviolet B, and oral corticosteroid mini‐pulse therapy for nonsegmental vitiligo: A retrospective study" was published in 2024. Journal: Skin Res Technol.

**TABLE 2:** Comparison of repigment grade in two groups during 3 months of treatment.

	Group			
Month	Case	Control	*Z*	*P*
First(MD)	1(1, 2)	1(1, 1)	−1.364	0.173
Second(MD)	2(1, 2)	1(1, 2)	−2.525	0.012*
Third(MD)	3(2, 3)	2(1, 3)	−2.773	0.006*

*Note*: *P*‐value < 0.05 considered as significant.

Abbreviation: MD, median.

**TABLE 3:** The number of patients with different grades in the two groups.

		Grade					
Month	Group	1	2	3	4	5	*P*
First(%)	Case	39(62.9)	22(35.4)	1(1.6)	0	0	0.173
	Control	42(76.3)	10(18.1)	2(3.6)	1(1.8)	0	
Second(%)	Case	16(25.8)	34(54.8)	9(19.5)	3(4.8)	0	0.012*
	Control	30(54.5)	16(29.0)	6(10.9)	3(5.4)	0	
Third(%)	Case	9(14.5)	20(32.2)	21(33.8)	8(12.9)	4(6.4)	0.006*
	Control	15(27.2)	26(47.2)	8(14.5)	3(5.4)	3(5.4)	

*Note*: *P*‐value < 0.05 considered as significant.

In the initial month, a significant proportion of patients in the treatment group demonstrated pigment deposition at grade 1 (62.9%) and grade 2 (35.4%). Conversely, the control group chiefly exhibited grade 1 pigment deposition (76.3%), with a solitary case progressing to grade 4. Nevertheless, during this month, the variations between the two groups did not attain statistical significance.

By the second month, the treatment group predominantly shifted to grade 2 (54.8%), whereas the control group advanced to grades 2 through 4. However, grade 1 remained dominant in the control group, constituting 54.5%. Significantly, from this juncture, the disparities in the treatment outcomes between the groups began to exhibit statistical significance.

During the evaluation conducted in the third month, the majority of the treatment group patients were observed to be at grades 2 and 3 (comprising 32.2 and 33.8%, respectively), with a minor fraction, 14.5%, still at grade 1. Conversely, 47.2% of the participants in the control group had recently transitioned to grade 2, while 27.2% continued to be at grade 1, engendering a progressively discernible statistical difference between the two groups. Figure 2 provides the dynamic transitions in pigment deposition grades throughout the 3‐month period.

**FIGURE 2:** The proportion of different grades in each group. *P*‐value < 0.05 considered as significant.

While the overarching trend appeared encouraging, the progress of individual patients fluctuated considerably each month. Specifically, in the case group, three patients (4.8%), and in the control group, two patients (3.6%) demonstrated repigmentation during the initial 2 months but experienced a plateau in the third month with no further progression.

The article "Combination of total glucosides of paeony, narrow‐band ultraviolet B, and oral corticosteroid mini‐pulse therapy for nonsegmental vitiligo: A retrospective study" was published in 2024. Journal: Skin Res Technol.

A subset of five patients (8.1%) from the case group and three patients (5.5%) from the control group displayed no significant change from the first to the second month but exhibited repigmentation in the third month.

A singular patient (1.6%) in the case group and three patients (5.5%) in the control group showed no further change after the first month of repigmentation.

Furthermore, two patients (3.2%) in the case group and three patients (5.5%) in the control group exhibited repigmentation during the first 2 months but regressed in the third, with an increase in the white spot area ranging from 5 to 10%.

Nevertheless, it is significant to note that every patient exhibited some degree of responsiveness to the treatments throughout the duration of the study.

Upon a more detailed examination of the correlation between degrees of improvement and demographic data, no significant associations were identified with variables such as gender, age, disease duration, clinical typing, or VASI scores. This result is shown in Table 4. In our endeavor to pinpoint the patients who would benefit most from TGP therapy, we conducted a meticulous analysis of the affected sites within the case group. This is shown in Table 5. This analysis underscored the heightened efficacy of treatments aimed at the head and neck regions in comparison to other areas, although no statistical variance in efficacy was noted amongst other body regions.

**TABLE 4:** The correlation between baseline information and degree of improvement in the two groups of patients.

Group	Month		Sex	Age	Course	Clinical typing	VASI
Case	First	*r*	0.095	0.195	0.076	−0.042	−0.051
		*P*	0.462	0.13	0.555	0.748	0.693
	Second	*r*	−0.035	−0.017	0.153	0.177	−0.203
		*P*	0.789	0.896	0.236	0.17	0.114
	Third	*r*	0.198	0.012	0.019	0.056	−0.172
		*P*	0.123	0.928	0.883	0.667	0.182
Control	First	*r*	−0.02	0.115	0.179	0.038	0.045
		*P*	0.884	0.402	0.19	0.785	0.744
	Second	*r*	−0.028	−0.047	0.02	−0.016	0.047
		*P*	0.839	0.732	0.884	0.91	0.733
	Third	*r*	−0.037	−0.071	0.167	−0.131	0.084
		*P*	0.79	0.606	0.222	0.342	0.541

*Note*: *P*‐value < 0.05 considered as significant.

**TABLE 5:** Comparison of the degree of improvement in different body parts in the case group.

	Body parts					
Month	Head and neck	Trunk	Limbs	General	*H*	*P*
First(MD)	2(1, 2)	1(1, 1)	1(1, 1)^a^	1.5(1, 2)	11.584	0.009*
Second(MD)	2(2, 3)	2(1, 2)^a^	2(1, 2)	2(1, 2)	11.802	0.008*
Third(MD)	3(3, 4)	2(1, 3)^a^	2(2, 3)^a^	2(2, 3)^a^	17.138	<0.001*

*Note*: *P*‐value < 0.05 considered as significant.

The article "Combination of total glucosides of paeony, narrow‐band ultraviolet B, and oral corticosteroid mini‐pulse therapy for nonsegmental vitiligo: A retrospective study" was published in 2024. Journal: Skin Res Technol.

Abbreviation: MD, median.

^a^ Compare with head and neck, *P* < 0.05.

A follow‐up commenced 6 months post‐treatment, facilitated through telephonic communication to ensure comprehensive patient outreach. All patients were subsequently asked to return to the hospital for an evaluation assessing vitiligo recurrence. Recurrence is defined as the reappearance or enlargement of the white spot area compared to the end of the last treatment. Table 6 revealed no statistical differences in recurrence rates between the two groups.

**TABLE 6:** Comparison of recurrence rates between the two groups.

	Recurrence			
Group	Yes	No	*X* ^2^	*P*
Case(%)	9 (14.5)	53 (85.5)	0.079	0.779
Control(%)	7 (12.7)	48 (87.3)		

*Note*: *P*‐value < 0.05 considered as significant.

Regarding side effects, five patients (8.1%) in the case group and four patients (7.3%) in the control group experienced gastrointestinal disturbances, these complaints included altered stool characteristics and increased frequency. Three patients (4.8%) in the case group and two patients (3.6%) in the control group developed itchy skin symptoms in the first month, but the symptoms disappeared in the following 2 months of evaluation. Notably, all reported symptoms were mild, thereby preventing any discontinuation of treatment due to these side effects. Complete blood count, biochemical tests, and plasma electrolyte tests were normal before and after treatment in both groups. Oxidative stress makers were analyzed as shown in Table 7. When comparing the case group before and after 3 months of treatment, SOD and MDA were significantly lower, while CAT, GPx, and GST were significantly higher, this was not found in the control group.

**TABLE 7:** Changes in oxidative stress makers before and after 3 months of treatment.

	Case group, mean ± SD			
	Before	After	*t*	*P*
SOD(U/mg)	3.69 ± 1.54	2.91 ± 1.36	2.979	0.003*
CAT(U/mg)	34.33 ± 2.68	36.71 ± 2.70	−4.927	<0.001*
GPx(U/mg)	1.73 ± 0.83	2.47 ± 0.82	−5.000	<0.001*
GST(UI/mL)	16.03 ± 3.55	20.66 ± 3.64	−7.180	<0.001*
MDA(mmol/mL)	5.65 ± 1.54	4.09 ± 1.50	5.725	<0.001*

	Control group, mean ± SD			
	Before	After	*t*	*P*
SOD(U/mg)	3.45 ± 1.33	3.50 ± 1.39	−0.151	0.880
CAT(U/mg)	34.82 ± 2.84	34.86 ± 3.10	−0.058	0.954
GPx(U/mg)	1.72 ± 0.44	1.76 ± 0.49	−0.457	0.649
GST(UI/mL)	17.81 ± 2.76	18.68 ± 2.41	−1.758	0.082
MDA(mmol/mL)	4.72 ± 1.78	4.54 ± 1.70	−0.528	0.598

*Note*: *P*‐value < 0.05 considered as significant.

Abbreviations: CAT, catalase; GPx, glutathione peroxidase; GST, glutathione‐S‐transferase; MDA, malondialdehyde; SD, standard deviation; SOD, superoxide dismutase.

The article "Combination of total glucosides of paeony, narrow‐band ultraviolet B, and oral corticosteroid mini‐pulse therapy for nonsegmental vitiligo: A retrospective study" was published in 2024. Journal: Skin Res Technol.

## 4 DISCUSSION

Within the realm of NSV therapeutic interventions, a range of approaches are pursued. In the context of TCM, scholars assert that vitiligo is analogous to “wind‐induced ailments” and indicative of “liver and kidney deficiencies.” Bai Shao, or white peony root, is believed to “balance qi and blood, dispel wind, and clear channels,” in addition to “nourishing the liver and kidneys,” thereby establishing it as a central remedy for vitiligo within traditional Chinese practices. Existing research by Yu et al. and Yuan et al. has illuminated the antioxidative stress mechanisms of TGP in preserving melanocytes.^7^, ^8^ Moreover, animal studies corroborate the capacity of paeoniflorin to enhance melanin synthesis and ameliorate vitiligo symptoms in mice.^9^ These insights accentuate the promising role of paeoniflorin in the treatment of vitiligo, thus advocating for extensive clinical research. Our study aimed to appraise the efficacy of TGP as a supplementary agent to the established OMP + NB‐UVB protocol in managing active NSV, while assessing its safety profile and its influence on recurrence rates.

Although theoretical investigations into TGP's role in vitiligo treatment are burgeoning, empirical studies remain limited. El Mofty et al. documented enhanced outcomes utilizing a combined OMP + NB‐UVB regimen for stable vitiligo compared to the application of either OMP or NB‐UVB singularly.^17^ Our study corroborates the efficacy of incorporating TGP into this regimen for the treatment of active NSV. A study by Jafarzadeh et al. systematically reviewed various studies of oral or injectable treatments for vitiligo and showed that different doses of OMP therapy produced significantly effective results.^21^ However the specific drugs used for OMP therapy are different in different literature and our study provides new insights into the addition of methylprednisolone to OMP therapy. In addition, they found that Methotrexate, Azathioprine, Cyclosporine, Mycophenolate mofetil, Simvastatin, Apremilast, Minocycline, Afamelanotide, Tofacitinib, Baricitinib, Antioxidants, and oral and injectable forms of CSs are all effective in the treatment of vitiligo, so future research directions should favor a comparison of the safety and efficacy of TGP in combination with these drugs.

Currently, there are no reported clinical studies pertaining to the application of TGP in vitiligo treatment. Beyond establishing the clinical advantages of TGP in this context, we are examining the specific phases during which it exhibits its effects, in order to furnish more nuanced usage guidelines. Our detailed analysis classified outcomes into five repigmentation categories, uncovering distinct variations over the 3‐month treatment period, as outlined in Table 2. Notably, although improvements were observed in both groups at the 1‐month interval, no significant disparity in efficacy was identified, potentially attributing to the brief initial period insufficient to evoke an optimal TGP response. Subsequent observations over 2 months substantiated this theory, showcasing a gradually expanding efficacy divide between the groups, with TGP's influence becoming notably evident between the second and third months. Encouragingly, by the third month, individual cases from both groups achieved grade 5 repigmentation, suggesting a potential for enhanced effects in the treatment group over extended durations. These findings imply that TGP yields gradual but sustained enhancements, rather than immediate benefits.

The article "Combination of total glucosides of paeony, narrow‐band ultraviolet B, and oral corticosteroid mini‐pulse therapy for nonsegmental vitiligo: A retrospective study" was published in 2024. Journal: Skin Res Technol.

Our site‐specific analysis underscored pronounced efficacy in treatments targeting the head and neck areas, echoing the conclusions of Lee et al.^20^ Their assessment of the synergistic efficacy of methylprednisolone pulse therapy and NB‐UVB for NSV demonstrated superior responses in the head and neck areas over a 3‐month span, paralleling our observations closely. However, their research did not distinctly ascertain whether these variances were derived from a 6‐month retrospective evaluation or from monthly clinical assessments. Our data, collected within the initial 2 months, revealed significant disparities in therapeutic efficacy between the limbs and trunk as compared to the head and neck regions. By the third month, the latter region exhibited markedly enhanced outcomes relative to the other areas. In summation, regardless of TGP incorporation, the consistent therapeutic responses established a reliable baseline, with corroborative findings across diverse research facilities offering persuasive evidence.

Previous reports have analyzed changes in oxidative stress markers in patients with vitiligo.^22^ Our study referred to these makers and performed a comparative analysis before and after treatment. Table 7 illustrates that SOD and MDA were significantly lower and CAT, GPx and GST were significantly higher in the case group patients after treatment, a change that was not seen in the control group. Yuan et al. had demonstrated that TGP was able to increase antioxidant enzyme activities in PIG1 and PIG3V cell lines by modulating the JNK/Nrf2/HO‐1 signaling pathway.^8^ And our findings demonstrate at the clinical level that TGP may benefit patients with vitiligo by reducing their oxidative stress levels. Notably, Li et al. investigated TanshinoneIIA, a compound extracted from the TCM Salvia miltiorrhiza. It reduces ROS levels and inhibits cellular pyroptosis by modulating the ROS/Nod‐like receptor protein 3 (NLRP3) signaling pathway in PIG1 and PIG3V cell lines.^23^ This implies that TGP and TanshinoneIIA act through different signaling modalities, so they likely have synergistic therapeutic potential.

The article "Combination of total glucosides of paeony, narrow‐band ultraviolet B, and oral corticosteroid mini‐pulse therapy for nonsegmental vitiligo: A retrospective study" was published in 2024. Journal: Skin Res Technol.

While TGP has been utilized in various clinical contexts, its safety within the realm of NSV treatment remained relatively unexplored prior to our investigation. Our preliminary data indicate a comparable safety profile between the TGP‐augmented regimen and traditional treatment modalities. Furthermore, there were no abnormal laboratory findings even after the treatment, only mild gastrointestinal symptoms and itchy skin symptoms were observed as side effects in both groups, a factor that did not inhibit ongoing medication use, thereby affirming its perceived safety. However, the side effect of itchy skin caused by NB‐UVB does have the potential to affect patient compliance. Platelet‐rich plasma (PRP) therapy is an emerging nonsurgical treatment modality, a systematic review and meta‐analysis of the treatment of vitiligo in a study by Wang et al. showed that the addition of PRP for combination therapy demonstrated better efficacy and higher patient satisfaction than carbon dioxide laser, excimer laser, and NB‐UVB therapy alone.^24^ Due to the favorable safety profile of TGP, combination therapy with TGP and PRP may achieve a lower incidence of side effects and produce better therapeutic outcomes.

The analogous relapse rates between the treatment and control groups suggest that TGP does not significantly impact NSV relapse prevention. Yet, given its noteworthy repigmentation rates accompanied by minimal side effects, extended TGP administration might reveal additional advantages.

Nonetheless, our study harbors several limitations. The limited sample size and the brief 3‐month treatment window may not fully encompass the broad therapeutic potential of TGP. Elongating the intervention duration, possibly to 6 months, might furnish a more nuanced understanding of its long‐term efficacy and safety. Additionally, owing to the dearth of double‐blinded randomized controlled trials (RCT), adopting more stringent methodologies could bolster the validity of future assessments. Noteworthy is that our analysis was confined to active NSV patients; delving into TGP's efficacy in cases of stable NSV could further elucidate its therapeutic scope.

## 5 CONCLUSION

In conclusion, our research accentuates the prospective advantages of incorporating TGP into the OMP + NB‐UVB treatment regimen for active NSV, specifically concerning lesions situated in the head and neck regions. We also demonstrated that TGP may act by reducing levels of oxidative stress. The favorable therapeutic results, combined with an acceptable safety profile and stable relapse rates, amplify TGP's potential as a supplemental NSV treatment strategy. This initiative, thus, lays a robust foundation for future large‐scale RCT, reinforcing the imperative for its inclusion in imminent clinical research endeavors to realize long‐term advancements.

The article "Combination of total glucosides of paeony, narrow‐band ultraviolet B, and oral corticosteroid mini‐pulse therapy for nonsegmental vitiligo: A retrospective study" was published in 2024. Journal: Skin Res Technol.

## CONFLICT OF INTEREST STATEMENT

The authors declare no conflicts of interest.

## Data Availability

The data that support the findings of this study are available on request from the corresponding author. The data are not publicly available due to privacy or ethical restrictions.
